# EEG-Controlled Wall-Crawling Cleaning Robot Using SSVEP-Based Brain-Computer Interface

**DOI:** 10.1155/2020/6968713

**Published:** 2020-01-11

**Authors:** Lei Shao, Longyu Zhang, Abdelkader Nasreddine Belkacem, Yiming Zhang, Xiaoqi Chen, Ji Li, Hongli Liu

**Affiliations:** ^1^Key Laboratory for Control Theory & Applications in Complicated Systems, Tianjin University of Technology, Tianjin 300384, China; ^2^Department of Computer and Network Engineering, College of Information Technology, United Arab Emirates University, Al Ain, P.O. Box 15551, UAE

## Abstract

The assistive, adaptive, and rehabilitative applications of EEG-based robot control and navigation are undergoing a major transformation in dimension as well as scope. Under the background of artificial intelligence, medical and nonmedical robots have rapidly developed and have gradually been applied to enhance the quality of people's lives. We focus on connecting the brain with a mobile home robot by translating brain signals to computer commands to build a brain-computer interface that may offer the promise of greatly enhancing the quality of life of disabled and able-bodied people by considerably improving their autonomy, mobility, and abilities. Several types of robots have been controlled using BCI systems to complete real-time simple and/or complicated tasks with high performances. In this paper, a new EEG-based intelligent teleoperation system was designed for a mobile wall-crawling cleaning robot. This robot uses crawler type instead of the traditional wheel type to be used for window or floor cleaning. For EEG-based system controlling the robot position to climb the wall and complete the tasks of cleaning, we extracted steady state visually evoked potential (SSVEP) from the collected electroencephalography (EEG) signal. The visual stimulation interface in the proposed SSVEP-based BCI was composed of four flicker pieces with different frequencies (e.g., 6 Hz, 7.5 Hz, 8.57 Hz, and 10 Hz). Seven subjects were able to smoothly control the movement directions of the cleaning robot by looking at the corresponding flicker using their brain activity. To solve the multiclass problem, thereby achieving the purpose of cleaning the wall within a short period, the canonical correlation analysis (CCA) classification algorithm had been used. Offline and online experiments were held to analyze/classify EEG signals and use them as real-time commands. The proposed system was efficient in the classification and control phases with an obtained accuracy of 89.92% and had an efficient response speed and timing with a bit rate of 22.23 bits/min. These results suggested that the proposed EEG-based clean robot system is promising for smart home control in terms of completing the tasks of cleaning the walls with efficiency, safety, and robustness.

## 1. Introduction

The idea of interfacing brains with machines/robots has long captured the human imagination. Brain-computer interface (BCI) technology intend to build an interface between the brain and any electrical/electronic device (e.g., a wheelchair, smart home appliances, and robotic devices) using electroencephalogram (EEG) which is a noninvasive technique for measuring electrical potentials from electrodes placed on the scalp produced by brain activity. Nowadays, the EEG technique has been used to establish portable synchronous and asynchronous controls for BCI applications. Noninvasive EEG-based BCIs are the most promising interface for space of applications for people with severe motor disabilities because of their noninvasiveness, low cost, practicality, portability, and being easy to use. For some disabled patients with physical disability or paralysis while the brain function is still normal, although they have a normal large brain consciousness and thought, they cannot communicate with the external environment through the severely damaged muscle and nervous system and complete the daily work independently. This has caused serious physical and mental trauma, and their lives are very painful, which will affect their recovery process to some extent. How to restore or enhance their control and communication capabilities to the outside world has been the goal that has been pursued for many years in the field of medical rehabilitation. Therefore, BCIs can be used for helping patients with severe brain disorders or muscle damages to regain their ability to communicate directly with the outside environment through the brain electrophysiology response [1–3]. BCI can also be beneficial for the elderly as advanced assistive and rehabilitative technologies and useful for young able-bodied for controlling video games for entertainment [4, 5] or controlling a robotic arm for several purposes [6–9]. However, most of the traditional brain-computer interface equipment is expensive, bulky, and tedious, which makes it difficult to popularize and apply brain-computer interface technology in real life. The portable brain-computer interface has become one of the hotspots in the field of the brain-computer interface because of its advantages of easy to carry, easy to use, safe, and reliable.

BCI technology is mainly divided into two types of brain activity measurement, invasive BCI, and noninvasive BCI, depending on the way of putting the electrodes to record the electrical brain activity [10–14]. Among them, the invasive BCI might lead to an immune reaction, which causes serious harm to the user, and it is hardly accepted by disabled people because of the invasiveness of the technique which requires a dedicated surgery, and its cost with equipment is very expensive and not covered by many governments yet. Although the noninvasive brain-computer interface is less accurate than the invasive BCI, it is still relatively cheaper compared with all other techniques and everyone can easily accept it. There are several paradigms to control machine or computer using our brain signal characteristics and the most popular ones are motor imagery [15, 16], P300 wave [17, 18], steady state visual evoked potentials (SSVEP) [19–21] for building practical brain-computer interface systems. So far, the SSVEP method was applied widely because of the high signal-to-noise ratio and robustness [22]. SSVEP induction means that when the human brain receives the stimulation of a fixed frequency scintillation block, an uninterrupted response related to the stimulation frequency will be generated in the visual cortex of the human brain. This SSVEP brain response is a very useful natural involuntary phenomenon which has been tested by researchers many times. The earliest SSVEP-BCI system, designed by Regan , in 1979, allowed subjects to select a flashing button on the computer screen by simply looking at the computer screen [23], basically achieving the desired design goals. Then, Mullerputz and Guneysu and Akin applied the SSVEP-BCI system to the physical control of neural limb and humanoid robot, respectively, and achieved good control results [24]. In this paper, we chose SSVEP because it does not need any training phase for subjects and has very high accuracy compared with P300 or motor imagery using single trial electroencephalography (EEG) signal. The commonly used signal processing and classification methods of SSVEP include fast Fourier transform (FFT), wavelet transform, canonical correlation analysis (CCA), linear discriminant analysis (LDA), and support vector machine (SVM). In this paper, CCA was used for developing our signal processing algorithm. Compared with other SSVEP signal classification algorithms [10–14, 25], CCA classification algorithm is fast, efficient, simple, and easy to use.

In some previous researches, the SSVEP paradigm was successfully used in writing tasks [26]. In the paper [27], we can see that the authors proposed a hybrid brain-computer interface system that combines P300 and SSVEP modalities. This combined system has improved the accuracy of EEG-based wheelchair control. In addition, SSVEP has been also used in the mental spelling system [28, 29]. In the paper [30], the authors used three flash speeds to control the small robot car. Lee et al. only use OZ as the reference electrode to collect and process EEG signals. In the paper [31], Lu and Bi have proposed a longitudinal control system for brain-controlled vehicles based on EEG signals. However, it is still unknown whether it can be used in the industry.

In this paper, a new type of intelligent crawler robot is designed for cleaning the walls, which is considered as one of the smart home appliances. Compared with the wheeled robot [32], the crawler robot has the advantages of long life and high carrying capacity. The intelligent crawling robot for the walls used in this experiment adds an adsorption device using negative vacuum pressure, which effectively solves the problem of sliding of the cleaning robot on a wall with a certain inclination angle. The BCI based on SSVEP can usually provide a high information transmission rate, the verification process of the system is relatively simple, and no training of the subjects is required. However, because the SSVEP of some subjects is very weak and vulnerable to the interference of other noise signals, how to accurately identify SSVEP from a short time window is still a challenging problem in BCI research based on SSVEP. This is also the subject that we will continue to study in the future. In this study, the SSVEP paradigm was designed to control the crawler robot for cleaning the dust on the walls. We used the high accuracy SSVEP paradigm to cooperate with our cleaning robot to complete the designed experiment. To our best knowledge, this is the first report, which used brain machine interface for crawling cleaning robot control to help persons with disabilities to improve their quality of life.

This paper is arranged as follows: in the Materials and Methods section, the experimental paradigm and analysis method of brain signal and the motion model of the intelligent crawling robot were introduced. At the same time, the offline experiment and online experiment are completed, and the data analysis is carried out. In the Results section, the offline and online experiments were summarized and discussed separately, and the accuracy and ITR of the experiment were obtained. Our experiments validate our views and achieve the desired results. In the Discussion part, we mainly talk about the limitations of the system and put forward the future changes. Finally, conclusion and prospects of future work are given in Section 5.

## 2. Materials and Methods

### 2.1. Participants and Experimental Paradigm

Seven healthy volunteers (4 males and 3 females, 23–27 years of age) were invited to join the experiment for performing some robot control tasks using their brain activity. None of the subjects have prior experience on brain-computer interfaces. Clear written informed consent was obtained from all the participants, who were informed in detail about the purpose and possible consequences of the experiment. The experimental protocol was carried out in accordance with the latest version of the Declaration of Helsinki.

The experiments were carried out in a quiet and comfortable environment to reduce the noise effect on our EEG recording. Subjects sat on a chair which is 60 cm away from the screen which contains the stimulation interface. In order to ensure the accuracy of the experiment, participants were required to avoid gnashing during the experiment. Because the SSVEP paradigm was easy to cause fatigue, the subjects can take a rest after one session. The flow of the experiment is shown in Figure 1. The experimental process is mainly divided into three parts. Firstly, the EEG acquisition device should be worn correctly for the subject and the subject's position should be adjusted. Secondly, the collected data are processed and classified by a signal processing computer. Finally, the processed instructions are sent to the lower computer, that is, the intelligent crawling robot.

### 2.2. Experimental Materials

As shown in Figure 1, the hardware system in this experiment mainly includes five parts: EEG signal acquisition system (Brain Products, Germany), computer for displaying visual stimulation interface, computer for signal processing, Bluetooth module for transmitting signals wirelessly, and intelligent crawling robot for cleaning dust on the walls.

We have avoided in this study to use EMOTIVE EPOC equipment which is relatively cheap consumer-grade EEG signal acquisition device because its measurement signal quality is not good enough for getting high classification accuracy using SSVEP modality. On the contrary, Brain Products can effectively collect the EEG signals induced by SSVEP, record real-time characteristic signals, and have good effects. EEG equipment (Brain Products) has the advantages of lightweight, flexible usage, and excellent and stable signals. Therefore, this EEG equipment was used to collect brain signals in our experiment. The EEG signal acquisition device used in our experiment is shown in Figure 2.

The EEG signal acquisition device selected in the experiment consists of 64 electrodes. 32 black circles represent effective electrodes and white circles are invalid electrodes. All 32 channel electrodes which include 30 EEG signals acquisition channels, 1 reference channel, and 1 ground channel were used to record brain signal. The position of each channel was shown by black circles. The sampling rate was 500 Hz. During the experiment, the impedance of each channel was always below 10 k ohms to ensure the quality of EEG signals. Because the SSVEP signal is generated by the visual cortex of the brain, the EEG signals of O1, O2, P7, and P8 channels near the visual cortex are collected in the experiment, which will not affect the acquisition of SSVEP signal, but also greatly reduce the amount of data processed by EEG.

The stimulation interface of the experimental paradigm was designed by using MATLAB psychology toolbox. This interface contains four blocks which flash at frequencies 6 Hz, 7.5 Hz, 8.57 Hz, and 10 Hz, respectively, four blocks were shown in the top, bottom, left, and right part of the screen, and the refresh rate of the screen was set in 60 Hz. The driving chip of the intelligent component used in the experiment is the L298P double H-bridge DC motor driving chip, which integrates most of the functions, making the chip more suitable for robot development. We designed a new crawler robot and also upgraded the adsorption capabilities of this robot. The traditional suction cup has a small adsorption capacity and is unstable, so the adsorption device we use uses a vacuum pump to generate a negative pressure to avoid the disadvantages of the conventional suction cup. Most of the photovoltaic robots on the market are roller brushes. The roller brushes are not only easy to absorb dust, but also occupy a relatively large area of the robot. Therefore, the crawling cleaning robot we use uses a three-legged brush head. After a series of experiments, the most suitable for the cleaning of the walls is to use a motor with a speed of 200 rpm to control our three-legged brush head. The robot relies on the suction cup to be adsorbed on the walls, and the walls can be stably and selectively cleaned, thereby reducing the trouble of cleaning the entire walls.

#### 2.2.1. Offline Experiment

The whole experiment was divided into offline and online subexperiments. Offline experiment was held to confirm the experiment set up and adjust the parameter for each subject. The offline experiment steps are as follows: start our stimulation interface, which starts with an exclamation mark to remind the subjects to start the experiment. After that the four different frequency blocks on the top, bottom, left, and right of the screen start to flicker. During the offline experiment, the subjects listened to the arrangement to look at each of the four different frequencies blocks. The subjects were assigned to look at each of the four scintillation blocks for five times, and the duration of each time was between 20 and 25 seconds. Twenty datasets were collected for each subject.

#### 2.2.2. Online Experiment

The experimental process of the subjects is shown in Figure 3. First, start our cleaning robot and turn on the cleaning device. Before the online experiment, we must ensure that the subject is in a comfortable position and that the EEG signal collection cap is correctly worn. Secondly, ensure that the cleaning robot is connected to our upper computer normally. In addition, the speed of the cleaning robot is set. After that, we started our online experiment. In the online experiment, the subjects confirm the position of the cleaning robot and the dirty place on the wall. Then, the subjects make the decision, which directs the clean robot to move and look at the responding flash block on the screen. At the same time, the EEG data were recorded from the participants; then it was analyzed at the host computer. The algorithm could recognize which block the subject looked at and transform the control command of the clean robot. Then, the command, which was recognized, was sent to the clean robot by the Bluetooth module. According to the command, the clean robot will move and make the walls cleaner.

To evaluate the experiment performance more easily, we set up several groups of online experiments. First, the clean robot was put on the wall, and the dirty place was not so far away from the original place of the clean robot. Therefore, the subjects can control the clean robot to reach the dirty place within 30 steps with optimized route, as shown in Figure 4.

This figure shows the path of a subject during an online experiment. For each session, the subject was limited to perform 30 steps. If the subject cannot control the clean robot to reach the destination, this experiment will finish and the task and system performance will be evaluated.

### 2.3. Signal Acquisition and Processing

The flowchart of signal acquisition and processing is shown in Figure 5. During our experiment, we used BrainVision Recorder software to record the EEG signals of the subjects. When using BrainVision Recorder software, we ensure that the impedance of the subjects' electrodes is below 10 k ohms. P7, P8, O1, and O2 channels, which cover the vision areas of the brain, were mainly analyzed.

Wavelet transform was employed as band-pass filter, removing DC Component of Signal. For SSVEP paradigm, canonical correlation analysis is a multivariate statistical analysis method that reflects the overall correlation between two groups of indicators by using the correlation between pairs of comprehensive variables; it has a good recognition effect in multichannel EEG signals. Compared with other SSVEP signal classification algorithms, CCA classification algorithm is fast, efficient, simple, and easy to use. In the paper [33], the CCA classification algorithm is compared with the power spectral density analysis (PSDA). The test results show that the classification accuracy of CCA classification algorithm is higher than that of PSDA. In the paper [34], the CCA classification algorithm is compared with the minimum energy combination (MEC), and the anti-interference ability of the CCA classification algorithm is found to be stronger. These results fully demonstrate the reliability of the CCA classification algorithm. Therefore, CCA is applied to the brain-computer interface system based on SSVEP. After preprocessing, CCA was used to analyze the brain signal.

One set of EEG signals is denoted as *x*(*t*), and the second set of signals *y*(*t*) is composed of signals with the same number of stimulation frequencies. We decompose a series of periodic signals into a series of Fourier functions. For a specific frequency *f*, there is the following equation

(1) $$\begin{array}{c} Y\left(f\right)=\left[\begin{array}{c} \sin\;2\;\pi fn\\ \cos\;2\;\pi fn\\ \sin\;4\;\pi fn\\ \cos\;4\;\pi fn\\ \cdots \\ \sin\;2N_{\text{h}}\pi fn\\ \cos\;2N_{\text{h}}\pi fn \end{array}\right],\\ n=\frac{1}{f_{\text{s}}},\frac{2}{f_{\text{s}}},\ldots ,\frac{N}{f_{\text{s}}}, \end{array}$$

where *N* is the number of sampling points. *f*_s_ is the sampling frequency, and *N*_h_ is the number of harmonics.

The feature extraction method of CCA is shown in Figure 6. Suppose that there are two groups of sample signals *X*=(*x*_1_,…, *x*_*n*_), *Y*=(*y*_1_,…, *y*_*m*_), and the linear combination of *x*=*X*^*T*^*W*_*x*_, *y*=*Y*^*T*^*W*_*y*_. Canonical correlation analysis method calculated the correlation *ρ*(*x*, *y*) between *x* and *y* under the condition that the coefficients *W*_*x*_ and *W*_*y*_ is maximum. The equation was shown as follows:

(2) $$\begin{array}{c} \underset{W_{x},W_{y}}{\max}\rho \left(x,y\right)=\frac{E\left[x^{T}y\right]}{\sqrt{E\left[x^{T}x\right]}E\left[y^{T}y\right]}=\frac{E\left[W_{x}^{T}XY^{T}W_{y}\right]}{\sqrt{E\left[W_{x}^{T}XX^{T}W_{x}\right]E\left[W_{y}^{T}YY^{T}W_{y}\right]}}. \end{array}$$

The correlation coefficient between the brain signal and four classes was computed. Therefore, the control command was set as the class with the maximum correlation coefficient.

In this study, information transmission rate (ITR) was calculated to evaluate the transmission performance of brain machine system. ITR (bit/min) can be calculated by the following formula:

(3) $$\begin{array}{c} \text{ITR}=\frac{60}{t}\left[{\text{log}}_{2}N+\text{Acc }\log_{2}\text{ Acc}+\left(1-\text{Acc}\right){\text{log}}_{2}\text{ Acc}\frac{1-\text{Acc}}{N-1}\right], \end{array}$$

where *t* represents the sampling time, Acc represents the correct rate, and *N* represents the number of classifications.

### 2.4. Motion Model Analysis of Intelligent Crawling Robot

The intelligent crawling robot we use communicates with the upper computer through the Bluetooth module. The speed of the cleaning robot can be set according to needs using Bluetooth serial port assistant. Among them, the running speed of the cleaning robot affects its turning angle. The turning motion model is as follows:

- We set a time parameter *t*; when *t* = 0, the robot is in the original position, assuming that the position of the cleaning robot coincides with the coordinate system {*X*, *O*, *Y*}, and the coordinates of the robot are {*X*_R0_, *O*_R0_, *Y*_R0_}, as shown in the blue position in Figure 7.
- After that, the robot performs a turning action. Where the time is *t*, the robot reaches a new position with coordinates of {*X*_R*t*_, *O*_R*t*_, *Y*_R*t*_}, as shown in the red position in Figure 7.

The whole turning process of the robot takes the origin as the center. For the turning motion of the robot, for any time *t*, we have the following:

(4) $$\begin{array}{c} \left\{\begin{array}{c} x\left(t\right)=\frac{1}{2}\int_{0}^{t}\left[v_{\text{L}}\left(t\right)+v_{\text{R}}\left(t\right)\right]\cos\left[\theta \left(t\right)\right]\text{d}t=0,\\ y\left(t\right)=\frac{1}{2}\int_{0}^{t}\left[v_{\text{L}}\left(t\right)+v_{\text{R}}\left(t\right)\right]\sin\left[\theta \left(t\right)\right]\text{d}t=0, \end{array}\right. \end{array}$$

where *ν*_L_ is the speed of the left wheel of the crawling robot, *ν*_R_ is the speed of the right wheel of the crawling robot, and *θ* represents the rotation angle of the crawling robot. We assume that *ν*_L_=−*ν*_R_; at this time, the crawling robot makes a rotation movement with the origin as the center, and the rotation angle is as follows:

(5) $$\begin{array}{c} \theta \left(t\right)=\frac{1}{D}\int_{0}^{t}\left[v_{\text{R}}\left(t\right)-v_{\text{L}}\left(t\right)\right]\text{d}t=\frac{2v_{R}}{D}t, \end{array}$$

where *D* is the distance between the two crawler wheels of the crawling robot.

## 3. Results

### 3.1. Offline Experiment and Result Analysis

For offline use, experiment data was saved in header file “.vhdr,” and EEGLAB toolbox was used to process the data. In order to achieve a good effect in our online experiment, we need to process the offline experiment data of different subjects and adjust the parameters. The CCA threshold divides the state of subjects into idle state and task state. By comparing the CCA correlation coefficient of the subject in the idle state with the CCA correlation coefficient in the task state, we can determine the threshold of each subject. We adjusted the subject threshold based on the analysis of the subjects' offline data, which were shown in Table 1.

### 3.2. Online Experiment and Result Analysis

In order to make our experimental data more accurate, when the subject completes the cleaning task within 30 steps, the time is stopped when the task is completed, but the subject continues to perform the task until the end of the 30 steps. When the subject does not complete the task within 30 steps, the time is counted based on the time when 30 steps are completed. Each subject has to perform six sets of tasks.

After the experiment, we performed some statistical analysis methods to evaluate the subjects' completion of the tasks. Four people were able to complete all the tasks with high accuracy and precision. The statistic results are shown in Table 1. The experimental data showed that the average accuracy of the subjects was 89.92 (with standard deviation of ±3.81%), and the ITR reached 22.23 ± 1.19 bits/min. The experimental situation of the subjects is shown in Table 2. In order to further verify the reliability of our experimental results and make the data statistically significant, we performed the variance calculation, and the variance calculation results are shown in Table 3. Accuracy in Table 3 is the average of the ratio of the total number of correct commands to the total number of commands in six experiments per person.

We noticed that our online experiments seem to have good output results compared to the existing BCIs in terms of task, accuracy, and ITR. We have listed the graphs for intuitive statistics and comparisons, as shown in Figure 8. These results show that our experiments validate our views and achieve the desired results.

## 4. Discussion

In this paper, EEG-controlled wall-crawling cleaning robot using SSVEP brain-computer interface is proposed, and the CCA algorithm is used for signal analysis. In this engineering study, the experiment results showed that our proposed brain-computer interface system is very promising and could control the proposed designed intelligent clean robot successfully to complete the cleaning tasks of a wall. The offline experiment provided the threshold for the next experiments. In addition, the test range of different experimenters can be determined by the same offline experiment. The online experiment was used to adjust the threshold to improve the classification accuracy of the experiment. After analyzing and calculating the data, we got the following results: the average accuracy of online experiment was 89.92%, and the ITR reached 22.23 bits/min. This shows that our experiments validate our research hypothesis and achieve the desired target. However, there are still some issues and limitations in the proposed BCI system.

The main innovation of this paper is to design a new type of cleaning robot that can enhance the abilities of the elderly users and help handicapped patients to control home appliances that might be available in their usual environment to increase their personal autonomy to be able to perform daily activities. Practicing EEG-based control in daily life might be a good option for enhancing brain abilities too. However, eye movements are also another option instead of using brain activity.

Electrooculography (EOG) is a technique for measuring the corneo-retinal standing potential that exists between the front and the back of the human eye. This technique has been widely used in developing human machine interfaces and it can be easily combined with brain activity. However, the signal of eye movements/blinking is relatively not weak. Therefore, it is difficult to remove this electrical interference due to the synchronization with EEG signal. If we use the eye movements directly to control the cleaning robot, we need to add eye gaze/tracking equipment, which needs to be well calibrated. In the process of eye movements' acquisition, the structure of the human eye leads to fatigue. In addition, the users are unable to look at the same target point for a long time. This long gaze concentration leads to the eye movements, the false eye jump, and the unconsciousness blinking [35]. These erroneous and unconscious EEG signals will bring difficulties to feature extraction and classification, resulting in a low recognition rate [36, 37].

In this paper, SSVEP is mainly used to overcome the shortcomings of using only eye movement instrument. Moreover, the combination of EEG and EOG (eye movement) as an innovative research for building hybrid BCIs is the direction of our future consideration.

After Hotelling put forward the typical classical algorithm in 1936, it has received great attention in various research fields. Some Japanese researchers adopted the canonical correlation analysis (CCA) method to extract two layers of reference signals from the actual SSVEP signal training concentration. Combining the obtained reference signals with CCA, an effective spatial filter for frequency recognition is derived, which greatly improves the recognition accuracy and information transmission rate of SSVEP [34]. Twelve categories of SSVEP signals were generated by modulating waveforms and were analyzed by CCA algorithm with an average accuracy of 92.31% [38]. Obviously, the application of CCA in EEG signal processing has been quite common, especially the frequency recognition of SSVEP signal which has high accuracy. In this paper, the traditional classical analysis algorithm is used. CCA algorithm is used to analyze SSVEP, the correlation coefficients between brain signal and four kinds of brain signal are extracted and calculated, and the transmission rate and the accuracy of online experiment are calculated. Although the CCA algorithm used in this paper has great advantages in SSVEP, compared with SVM method [25], it still needs to be improved. Because the human brain has complex neural mechanisms, it may not be a simple linear transformation in the transmission of electrical signals in the brain. In addition to the time and frequency characteristics that we usually consider, EEG also contains other important data characteristics, such as the variability between experiments and the specificity between subjects [12, 39]. Therefore, improving feature extraction and classification algorithm will be the focus of our future research to improve the robustness and accuracy of the system and reduce errors.

## 5. Conclusion

In this paper, we proposed a new experimental paradigm for EEG-based clean robot control, which extended the usage of brain-computer interface. Compared with other paradigms like motor imager and P300, SSVEP is better for real-time application because SSVEP-based paradigm is not a subject-specific BCI, which requires individual data calibration regularly and system training, and it has achieved higher accuracy across subjects. For different subjects, the corresponding conditions are also different. During the experiment, we have selected the appropriate EEG acquisition cap according to different subjects. In addition, the fatigue issue was clearly observed in some subjects. Therefore, we eliminated the inaccurate experimental data caused. Although the conditions of different subjects are different, we also verified our system through our experiments.

Noninvasive brain-computer interface technology has built a bridge between human brain and smart robots, which has important research significance. In the near future, daily life BCI applications will be involved in fields that are more new. With the development of science and technology, brain-computer interface technology will not only bring hope to people with disabilities, but will also be more integrated into the life of ordinary people, bringing more convenience and use to our life. Through this experiment, we hope that in the future, we can recruit more subjects to verify the proposed system and make complex system in different conditions such as controlling a swarm of cleaning robots by one operator brain only.

## Figures and Tables

**Figure 1:** Experimental flowchart for our proposed SSVEP EEG-based BCI for robot control system.

**Figure 2:** EEG electrodes placement used in our experiment using Brain Products equipment.

**Figure 3:** Flowchart of the subject performing a brain control task.

**Figure 4:** The online experimental paradigm with respect to the path of a representative subject.

**Figure 5:** Signal analysis and processing steps of the proposed algorithm for decoding SSVEP from the EEG signal.

**Figure 6:** Feature extraction phase of CCA.

**Figure 7:** Moving model of the crawler robot turning.

**Figure 8:** Experimental results of our proposed BCI system for evaluating the classification accuracies, ITR, and variance value among subjects. (a) The classification accuracy for each subject. (b) Information transfer rate for each subject. (c) Variance value for each subject.

**Table 1:** Coefficients for different SSVEP states.

SSVEP state	Mean ± SD
6 Hz	0.40 ± 0.12
7.5 Hz	0.44 ± 0.09
8.57 Hz	0.50 ± 0.10
10 Hz	0.51 ± 0.05
Idle	0.16 ± 0.04

**Table 2:** Experimental statistics.

Subject	Number of completed tasks	The average time
S1	6	6′25″
S2	6	6′56″
S3	6	6′17″
S4	6	5′59″
S5	4	6′00″
S6	5	6′56″
S7	4	7′00″

**Table 3:** Data statistics of subjects.

Subject	Accuracy (%)	ITR (bits/min)	Variance
S1	91.11	22.52	9.88
S2	89.45	22.26	12.65
S3	91.11	22.52	6.16
S4	91.11	22.52	9.88
S5	91.67	22.61	13.89
S6	88.89	22.17	13.57
S7	86.11	21.04	5.25
Average	89.92 ± 3.81	22.23 ± 1.19	10.18 ± 4.93

## Data Availability

The datasets generated and analyzed during the current study are not publicly available due to Tianjin University of Technology policy but are available from the first author upon reasonable request.
